The article "Cardioprotective Effect of Danshensu against Ischemic/Reperfusion Injury via c-Subunit of ATP Synthase Inhibition" was published in 2017. Journal: Evid Based Complement Alternat Med.

# Cardioprotective Effect of Danshensu against Ischemic/Reperfusion Injury via c-Subunit of ATP Synthase Inhibition

**DOI:** 10.1155/2017/7986184

**Published:** 2017-11-08

**Authors:** Qing Gao, JingYi Zhao, Zixuan Fan, Jiadi Bao, Dawei Sun, Huhu Li, Chun Sun, Xijuan Jiang

**Affiliations:** School of Integrative Medicine, Tianjin University of Traditional Chinese Medicine, Tianjin 300193, China

## Abstract

Mitochondrial permeability transition pore (MPTP) opening is the main culprit of ischemic/reperfusion (IR) injury. It is reported that c-subunit of ATP synthase is the core component of MPTP. Danshensu (DSS), a monomer isolated from the traditional Chinese herb Danshen, has showed cardioprotective effect against IR injury through unknown mechanism. In this study, rat hearts were suspended in Langendorff instrument and perfused with Krebs-Henseleit (KH) buffer containing DSS for 60 minutes, followed by 30 minutes of global ischemia. Parameters including heart rate, left ventricular developed pressure, and the rate of left ventricle diastolic pressure change were recorded to assess their cardiac function. All these indexes were improved in DSS group. The rate of cardiomyocytes apoptosis and MPTP opening were both inhibited in DSS group. In addition, DSS administration leads to downregulation of c-subunit of ATP synthase in both mRNA and protein levels. Consistently, when c-subunit of ATP synthase was overexpressed in H9C2 cells through pcDNA3/5G1 plasmid transfection, MPTP opening was enhanced when the cardioprotective effect of DSS also tapers. In conclusion, DSS could alleviate cardiac IR injury via inhibiting c-subunit of ATP synthase expression.

## 1. Introduction

Although routine treatments for cardiac ischemia such as coronary bypass surgery, thrombolysis, and percutaneous coronary intervention have made satisfying outcome, the occurrence of ischemic/reperfusion (IR) injury should not be neglected [1]. Multiple reasons, such as oxidative stress, inflammation, and cell death, contribute to IR injury. Recent studies showed that mitochondrial permeability transition pore (MPTP) opening is the fundamental cause of IR injury [2]. MPTP is a nonspecific pore at the inner mitochondrial membrane whose opening is triggered by Ca^2+^ overload or oxidative stress. MPTP opening is a process that its inner membrane suddenly enables free diffusion of solutes up to 1.5 kDa in size [3]. However, excessive MPTP opening will lead to inner membrane potential collapse, respiratory chain uncoupling, and halt of mitochondrial ATP synthesis. Eventually mitochondria become swelling and rupture and ensue with cell death [4]. Taking into consideration its role in reperfusion-mediated cardiac damage, MPTP opening is a prime target for therapies that aims at cardioprotection [5].

The article "Cardioprotective Effect of Danshensu against Ischemic/Reperfusion Injury via c-Subunit of ATP Synthase Inhibition" was published in 2017. Journal: Evid Based Complement Alternat Med.

MPTP is considered to be a multiprotein complex includes the voltage-dependent anion channel at the outer membrane, adenine nucleotide translocator at the inner membrane, and cyclophilin D at the matrix [6, 7], all of which are considered to be major modulators of MPTP. However, they are dispensable to the structure of MPTP [8, 9]. Recent studies showed that c-subunit of the F_0_ ATP synthase constitute a critical component of MPTP [10, 11]. Multiple copies of c-subunit form a closed ring, which forms the ion-driven membrane rotors of ATP synthases. The c-subunit comprises two trans-membrane helices, and its c-ring features an ion-binding site in paired adjacent subunits. Normally, the c-ring remains closed until the episode of Ca^2+^ overload or oxidative stress such as during IR process when it opens followed by opening of MPTP [12]. In contrast, He et al. reported persistence of MPTP opening in the absence of subunit c of human ATP synthase [13]. The c-ring model of MPTP meets challenges. Although we cannot make sure whether c-subunit is the core of MPTP, altered c-ring of ATP synthase increases sensitivity of mitochondria to undergo MPTP opening as important determinants of the reduced tolerance to ischemic-reperfusion injury [14]. Therefore, inhibition of extravagant opening of c-ring could inhibit extravagant opening of MPTP.

Danshen is an herb medicine used in clinic to treat cardiovascular diseases, such as myocardial hypertrophy and ischemia reperfusion injury. Danshensu (DSS) is a major water-soluble active component of Danshen. The mechanism of DSS in treating IR is known to be through its antioxidants effect and ability to reduce Ca^2+^ overload [15–17]. Therefore, we proposed DSS might play a role in preventing the opening of MPTP. In the present study, we investigated the role of DSS in treating IR through manipulating the expression of c-ring of ATP synthase.

## 2. Materials and Methods

### 2.1. Drugs and Regents

DSS was provided by National Institutes for Food and Control, of purity of over 98%. Cell Counting Kit-8 (CCK-8) kit was purchased from Dojindo (Rockville, MD, USA). Terminal-deoxynucleotidyl transferase mediated nick end labeling (TUNEL) kit was brought from Roche (St Louis, MO, USA). Mitochondria Isolation Kit was purchased from Beyotime Biotechnology Inc. (Beijing, China). MPTP kit (For mitochondrial and cell use) was purchased from GENMED (Shanghai, China). Tetrachloro-tetraethyl benzimidazole carbocyanine iodide (JC-1) was purchased from Invitrogen (Thermo Fisher, Shanghai, China). Primary antibody against c-subunit and caspase-3 were purchased from Abcam (Cambridge, UK). Quantitative polymerase chain reaction (QPCR) kit was from Tiangen (Beijing, China). Plasmid was purchased from GeneChem (Shanghai, China).

The article "Cardioprotective Effect of Danshensu against Ischemic/Reperfusion Injury via c-Subunit of ATP Synthase Inhibition" was published in 2017. Journal: Evid Based Complement Alternat Med.

### 2.2. Animals

Male Sprague-Dawley (SD) rats (250 ± 30 g) were supplied by Experimental Animal Center of the Tianjin University of Traditional Chinese Medicine. Rats (*n* = 45) were randomly assigned to the following groups: control group, model group, and DSS group with 15 rats in each group. All procedures conform to the regulations that was stipulated by Animal Care Committee of Tianjin University of Traditional Chinese Medicine and to the Principles of Laboratory Animal Care that were formulated by the National Society for Medical Research and to the Guide for the Care and Use of Laboratory Animals that was published by the National Institute of Health (NIH Publication number 85-23, revised 1996).

### 2.3. Langendorff Isolated Heart Perfusion Preparation

The rats were anesthetized by chloral hydrate (300 mg/kg, ip). As soon as negative tail-flick response was confirmed, its chest was opened. The heart was rapidly harvested and then incubated in ice-cold Krebs-Henseleit (KH) buffer with aorta cannulated. Following Langendorff method, the heart was mounted on Langendorff apparatus and retrogradely perfused* in vitro* via aorta at the pressure of 70 mmHg. The perfusion medium was continuously bubbled with a mixture of 95%  O_2_ and 5%  CO_2_ at 37°C, reaching the pH of 7.4. Each heart was housed in a controlled heart chamber maintained at 37°C. Coronary perfusion was applied by Langendorff system using KH buffer, containing 105.7 mM NaCl, 5.36 mM KCl, 1.28 mM CaCl_2_, 1.084 mM MgCl_2_, 6 mM H_2_O, 1.18 mM KH_2_PO_4_, 18 mM NaHCO_3_, and 11 mM Glucose. Control group was reperfused with KH continuously. In model and DSS groups, perfusion was stopped for 30 mins followed by reperfusion for 60 min. DSS at 10 *μ*M [18] was added to KH solution in the DSS group (Figure 1). Then the heart tissues were used for the next experiments.

### 2.4. Cell Culture and Treatments

H9C2 cell line isolated from rats was used in our study. ATP5G1-overexpression plasmid was transfected by lipo2000 into H9C2 cell. The transfect efficiency was assessed by QPCR after 24 h. Oxygen glucose deprivation (OGD) model was used to simulate ischemic-reperfusion injury. In detail, cells were replaced with nonglucose Dulbecco's modified eagle medium (DMEM) and incubated in 95%  N_2_, 5%  CO_2_ atmosphere for three hours; then the cells were replaced with high-glucose DMEM containing 10%  FBS in 95%  O_2_, 5%  CO_2_ for four hours.

Cells were divided into five groups: control, model, DSS, pcDNA3/5G1, and pcDNA3/5G1 + DSS group. In DSS and DSS + 5G1 group, 10 *μ*M DSS in the reoxygenation step was added. Cell viability, apoptosis, and MPTP opening status were detected by CCK-8 kit, TUNEL staining, and cell MPTP kit, respectively.

The article "Cardioprotective Effect of Danshensu against Ischemic/Reperfusion Injury via c-Subunit of ATP Synthase Inhibition" was published in 2017. Journal: Evid Based Complement Alternat Med.

### 2.5. Cardiac Function Measurement and Observation

Cardiac function was evaluated by parameters including left ventricular developed pressure (LVDP), the max and minimum rate of left ventricle diastolic pressure change per min (±dp/dt), and heart rates (HR). LVDP equals left ventricle end systolic pressure minus by left ventricle end diastolic pressure. ±dp/dt max is the maximal and minimum rate of pressure development. LVDP, ±dp/dt max, and HR were calculated from the LV pressure curve. These parameters were recorded continuously using Powerlab data acquisition system (8SP Chart 5 software; A.D. Instruments, Castle Hill, Australia) [19]. Part of left ventricular tissues were harvested and stored as frozen section for further TUNEL examination. Mitochondria isolated from heart tissue were used for MPTP opening and mitochondrial membrane potential (MMP) analysis. The remaining heart tissues were homogenate at 10% (w/v) and stored at −80°C for further quantifying c-subunit mRNA level and ATP synthase protein level.

### 2.6. TUNEL Examination

Terminal-deoxynucleotidyl transferase mediated nick end labeling (TUNEL) assay was used to evaluate apoptosis in ischemic reperfused heart tissue and H9C2 cell. Rat hearts were harvested and frozen-sectioned which were then processed under instruction of In Situ Cell Death Detection Kit, Fluorescein (Roche). For quantitative analysis, TUNEL-positive cells in five different slides from different hearts were counted. The apoptotic index was defined as the percentage of TUNEL-positive myocytes per slide.

### 2.7. MPTP Opening and MMP Detection

For* in vivo* study, mitochondria were isolated from heart tissue according to the protocol of Mitochondria Isolation Kit [20]. MPTP opening and mitochondrial membrane potential were then examined under instruction of Mitochondria MPTP fluorescence detection kit (For mitochondria use only) and tetrechloro-tetraethylbenzimidazol carbocyanine iodide (JC-1) [21]. For* in vitro* study, MPTP opening was detected using cell MPTP fluorescence detection kit (For cell use only).

### 2.8. Quantitative Polymerase Chain Reaction (QPCR)

Total RNA was isolated from the cardiac tissue using Trizol (invotrogen) and reversely transcribed into cDNA by superscript reverse transcriptase (Tiangen, Beijing, China) at 42°C for 1 h. Reverse transcription material (100 ng) was amplified with Taq DNA polymerase (Tiangen, Beijing, China). Primers were synthesized by Sangon Biotech (Shanghai, China).

The article "Cardioprotective Effect of Danshensu against Ischemic/Reperfusion Injury via c-Subunit of ATP Synthase Inhibition" was published in 2017. Journal: Evid Based Complement Alternat Med.

The primer pair specific to ATP 5G1 is as follows:

  Forward sequence 5′-GGAGTGGGAGTGCAGATTGAA-3′
  Reverse sequence 5′-TGGTACAGGAGCGGATCAGA -3′

The primer pair specific to GAPDH is as follows:

  Forward sequence 5′-GCATCTTCTTGTGCAGTGCC-3′
  Reverse sequence 5′-GATGGTGATGGGTTTCCCGT -3′

Polymerase chain reaction (PCR) products of LOX-1 and GAPDH were 78 base pairs and 262 base pairs, respectively. Forty cycles (94°C for 30 s; 60°C for 1 min; and 72°C for 1 min) were used in PCR reaction. Gene expression profile was analyzed by 2^−ΔΔCT^ ([delta] [delta] CT ) method.

### 2.9. Western Blotting

Proteins were obtained from heart tissues after the whole perfusion process. Quantification of the protein was conducted using a modified bicinchoninic acid (BCA) assay (Cwbio, China). Protein samples were prepared by homogenizing rat heart, then being boiled for 5 minutes with loading buffer (Cwbio, China). Samples were separated using sodium dodecyl sulfate polyacrylamide gel electrophoresis (SDS-PAGE) on 15% gel and transferred onto polyvinylidene fluoride (PVDF) membrane by electroblotting. After being blocked using skimmed milk for 1 h, the membranes were incubated at 4°C overnight with the primary antibody. The following day, the membranes were washed and incubated with the goat anti-rabbit horseradish peroxidase-conjugated secondary antibody at room temperature for 1 h. Protein bands were visualized using an enhanced chemiluminescence kit (Cwbio, China) under a ChemiDoc imaging system (Bio-Rad Laboratories, Berkeley, CA, USA).

### 2.10. Statistical Analysis

Each quantitative experiment was repeated three times. Statistical results were presented as means ± SEM. *P* values of <0.05 were denoted as statistically significant. One-way analysis of variance (ANOVA) was used to assess the differences among the groups. Fisher's least significant difference (LSD) was used in multiple comparisons between groups. Nonparametric statistical method of Mann–Whitney test was used to assess histopathology of myocardial damage level data. All statistical analyses were calculated using SPSS 17.0 (International Business Machines Corp., Armonk, NY, USA).

## 3. Results

### 3.1. Effect of DSS on Cardiac Function and Cardiomyocytes Apoptosis

The hearts were harvested from rats and then hung in the Langendorff apparatus. Cardiac function was recorded by the Powerlab/16s record software in Langendorff system through the whole reperfusion process. Control group was perfused with KH buffer for 120 min. For model and DSS group, first perfusion for 30 min, then through 30 min ischemia, and 60 min reperfusion: 10 *μ*M DSS was added to KH buffer in the DSS group during reperfusion step. The normal HR was within 250–300 BPM. During ischemia, HR declined rapidly to zero. HR was not recovered following reperfusion for 60 min in model group. On the other side, in DSS group, HR recovered to normal level after reperfusion for 20 min. In control group, LVDP was maintained constantly at 50–80 mmHg. In model group, it was kept at 20–30 mmHg in the reperfusion process On the contrary, LVDP recovered to normal level when heart undergoing reperfusion for 20 min in DSS group. Similarly, ±dp/dt index failed to recover to baseline in model group during the whole reperfusion process while it recovered to normal level when heart was reperfused for 20 min in the DSS group (Figure 2). These results indicated that DSS could improve cardiac function significantly in ischemic-reperfusion process.

The article "Cardioprotective Effect of Danshensu against Ischemic/Reperfusion Injury via c-Subunit of ATP Synthase Inhibition" was published in 2017. Journal: Evid Based Complement Alternat Med.

Cardiomyocytes apoptosis was detected by TUNEL method and caspase-3 expression. As shown in Figures 3(a) and 3(b), cell apoptosis rate in model group was 3 times over the DSS group. As shown in Figures 3(c) and 3(d), caspase-3 expression in heart of model group was 2 times higher than the DSS group, which means DSS can alleviate cell apoptosis.

### 3.2. Effect of DSS on the Opening of MPTP

When the reperfusion process finished, hearts samples were harvested. Mitochondria were isolated from heart tissue for MPTP opening detection. Mitochondria MPTP kit and JC-1 dye were used to evaluate the status of MPTP opening. Mitochondria MPTP kit used calcein-AM as fluorescence probe. When calcein-AM entered into mitochondria, it was excised by lactonase to produce fluorescent calcein with strong polarity and then captured by mitochondria. At the same time, calcein outside mitochondria was quenched by cobalt ions. As soon as MPTP opens, calcein release from mitochondria can also be quenched by cobalt ions. Thus the relative fluorescence unit (RFU) changes in the mitochondria indicate MPTP opening.

MPTP opening in model group significantly enhanced compared to its intact level in DSS group. JC-1 was used to detect the mitochondrial membrane potential (MMP) changes, which reflect the degree of MPTP opening indirectly. Our results showed that MMP decreased significantly due to IR in model group compared to its unaltered level in DSS group (Figure 4). In a word, DSS can inhibit the MPTP opening.

### 3.3. Effect of DSS on the Expression of ATP c-Subunit

Total protein was obtained from heart tissue after the reperfusion process. C-subunit of ATP synthase expression in heart tissue was detected by western blotting. Expression of ATP c-subunit was significantly upregulated after IR while it remained in normal level in DSS group (Figure 5). The results indicated that DSS inhibited MPTP opening possibly through inhibiting c-subunit of ATP synthase expression.

The article "Cardioprotective Effect of Danshensu against Ischemic/Reperfusion Injury via c-Subunit of ATP Synthase Inhibition" was published in 2017. Journal: Evid Based Complement Alternat Med.

### 3.4. Effect of DSS in ATP c-Subunit Overexpressed H9C2 Cell Lines

H9C2 cells were transfected with pcDNA3/5G1 plasmid. To evaluate the transfection effect, both mRNA transcription level and protein expression level of ATP 5G1 were quantified. ATP 5G1 mRNA expression was four times higher than that of the nontransfection cell (Figure 6(a)). Consistently, ATP5G1 protein expression level was shown to be three times higher than that of nontransfection cell.

DSS was also shown to be able to improve cell vitality as indicated by CCK8 in all group but not in the pcDNA3/5G1 transfection group (Figure 6(d)). ATP 5G1 mRNA expression was upregulated in model group but not in DSS group, which insinuated that DSS can inhibit ATP 5G1 mRNA expression during IR injury (Figure 6(e)). DSS was also shown to be able to protect cells from apoptosis in control H9C2 cells but not in the plasmid transfection cells (Figure 7). MPTP opening was also inhibited in control cells but not in the plasmid transfection group (Figure 6(f)). Therefore, DSS could protect cells from ischemic-reperfusion injury through inhibiting c-subunit of ATP synthase expression, and the protection effect waned under circumstance of ATP 5G1 overexpression.

## 4. Discussion

MPTP opening plays a critical role during the episode of cardiac ischemic-reperfusion injury. The c-subunit of ATP synthase was used as target for new drug development [22]. Being a component in Chinese herb that was used widely in cardiovascular diseases, the underlying mechanism of DSS in treating IR injury still needs to be elucidated.

DSS, a water soluble isolated from* Salvia miltiorrhiza* (Danshen), has been widely used in clinic for the treatment of ischemic-reperfusion injury in China [23]. Several studies reported its effects in improving cardiac function both* in vivo* and* in vitro*, which are consistent with our results [15]. In this study, DSS improve cardiac function indicated by the fact that HR and LVDP were both upregulated significantly but were recovered soon after reperfusion in DSS group. What is more, it was shown that apoptosis rate declined significantly in DSS group followed IR injury both* in vivo* and* in vitro*. DSS could improve cell viability and decrease cell apoptosis rate in the OGD model.

Many studies explore the underlying mechanism of DSS in alleviating IR injury, such as its antioxidant and antiapoptotic effect and its role in reducing the calcium overload [16, 17, 24], but no study has reported its role in MPTP opening under IR injury background. Previous studies revealed that MPTP opening is the main cause of cell death and cardiac damage [25]. MPTP has been considered as nonspecific pores, whose opening is responsible for the osmotic influx of water into the mitochondrial matrix and results in swelling of mitochondria and dissipation of the mitochondrial membrane potential with cell death ensuring [17]. Results showed that the degree of MPTP opening was upregulated with decreased MMP during IR. On the contrary, the degree of MPTP opening declined and MMP remains normal level with DSS treatment in episode of IR. Not surprisingly, the inhibition effect of DSS on MPTP opening was confirmed* in vitro *too.

The article "Cardioprotective Effect of Danshensu against Ischemic/Reperfusion Injury via c-Subunit of ATP Synthase Inhibition" was published in 2017. Journal: Evid Based Complement Alternat Med.

As nonspecific pores, the exact components of MPTP are not fully understood. Although MPTP is modulated by cyclophilin D, Voltage-Dependent Anion Channel (VDAC), and Phosphate Carrier [25–27], recent studies found that the main modulate component of MPTP is the c-ring of ATP synthase, the number of which was determined by the expression of c-subunit [11, 12, 28]. The ring of c-subunits constitutes the membrane domain which were shared by both MPTP and ATP synthase. Azarashvili et al. [29] demonstrated that MPTP formation is associated with de novo assembly of channels comprising c-subunit, polyhydroxybutyrate, and inorganic polyphosphate, which is independent of ATP synthase. By contrast, He et al. found persistence of the mitochondrial permeability transition in the absence of subunit c of human ATP synthase [13]. C-subunit knockout human HAP1 and 143B cells preserves the characteristic properties of the permeability transition pore. Given in the opposite results obtained from 293T cells and rat cortical neurons [12, 25], whether c-subunit is the component of MPTP in human cells and whether c-subunit knockout cells have alternative means to develop permeability still needed to be further researched.

In the present study, our results showed that c-subunit of ATP synthase was downregulated with DSS treatment under IR scenario both* in vivo* and* in vitro*. This indicates that inhibition of c-subunit expression can alleviate IR injury. Regardless of the relationship between c-subunit and MPTP, c-subunit is the potential target to treat IR.

ATP subunit has three isoforms, encoded by ATP5G1, ATP5G2, and ATP5G3 genes, respectively [25]. Mammalian c-subunit consists of a mature protein with 76 amino acids, which is identical between all three isoforms. All these three c-subunit isoforms are functional and contribute to the F_0_ structure, but they have variable expression patterns in different tissues. For example, ATP 5G1 was abundantly expressed in heart [30].

Cardiomyocytes are sensitive to the changes of microenvironment, especially ischemia. Numerous studies have reported that mRNA transcription and protein expression change during the first 90 minutes of ischemic-reperfusion episode in both human and animals [31, 32]. ATP 5G1, which target to mitochondria, can be imported into mitochondria under ischemic conditions [10, 29].

The article "Cardioprotective Effect of Danshensu against Ischemic/Reperfusion Injury via c-Subunit of ATP Synthase Inhibition" was published in 2017. Journal: Evid Based Complement Alternat Med.

*In vitro* experiment shows that the cardioprotective effect of DSS disappeared under circumstance of ATP 5G1 overexpression cells. These results suggested that the effect of DSS might be through regulating ATP 5G1 gene expression. However, our study had limitations that the specific pathway related to ATP 5G1 needs to be further investigated. Also, the respiratory activity of the DSS-treated mitochondria should also be evaluated; it has been suggested that mitochondria may be less leaky to protons in the absence of the c-subunit [13]. In addition, excessive c-subunit will form hydrophobic aggregates (such as in Batten disease) that increase mitochondrial coupling of oxygen [33]. Therefore, it is interesting to know whether reduction of c-subunit expression improves the mitochondrial ATP bioenergetics.

There are also studies that support the role of c-subunit in MI treatment. Campo et al. enrolled 158 patients with first episode of acute anterior ST-segment elevation myocardial infarction (STEMI) who were treated successfully with percutaneous coronary intervention (PCI) [34]. They provided the first evidence that c-subunit is detectable in the serum of STEMI patients, but the data did not follow normal distribution (median 6.3% [4–9.3%]; range 1.1–47.5%). In humans, the roles of MPTP and c-subunit are strongly influenced by several confounding factors, including thrombolysis application in myocardial infarction, myocardial perfusion grade, thrombolysis in myocardial infraction (TIMI) frame court, extent of ST-segment resolution, and presence of cardiac marker. These findings help us to explain why drugs to treat reperfusion injury always failed in randomized clinical trials.

## 5. Prospective

Herein, DSS was shown both* in vivo* and* in vitro* that can protect cardiomyocytes from apoptosis and inhibit MPTP opening in IR injury. Expression of c-subunit of ATP synthase was demonstrated to decline in both mRNA and protein level with DSS administration in IR background. The protection effect of DSS recedes with ATP 5G1 overexpression, which indicates its role in DSS signaling.

The limitation of the present study needs to be improved in the future research. Firstly, the drug effect on subunit c might be mediated by an effect on the whole ATP complex. Whether DSS can alter other subunits of ATP synthase is not clear at present. In addition, the underlying mechanism of the curative effect of DSS is related to inhibition of c-subunit expression which needs to be confirmed in human.

The article "Cardioprotective Effect of Danshensu against Ischemic/Reperfusion Injury via c-Subunit of ATP Synthase Inhibition" was published in 2017. Journal: Evid Based Complement Alternat Med.

## Figures and Tables

**Figure 1:** *Scheme of IR experiment*. The hearts were harvested from rats and then hung in the Langendorff apparatus. Control group was perfused with KH buffer for 120 min. Model and DSS group first perfusion for 30 min, then through 30 min ischemia, and 60 min reperfusion: 10 *μ*M DSS were added to KH buffer in the DSS group during reperfusion step.

**Figure 2:** *Cardiac function data recorded by Powerlab/16s software*. After the hearts were hung in the Langendorff apparatus, Powerlab/16s software was used to collection the data of cardiac function. (a) Heart rate. (b) Left ventricular developed pressure (LVDP). (c) Development of left ventricular pressure maximum rising rate (+dp/dt). (d) Development of left ventricular pressure minimum decline rate (−dp/dt). Values were expressed as mean ± SEM. ^*∗*^*P* < 0.05, compared to control group.

**Figure 3:** *Cardiac apoptosis rate assay*. (a) TUNEL detection. Nuclear was stained by DAPI and presents blue fluorescent in heart tissue. Apoptosis was detected by DNA strand breaks stained by TUNEL kit and present green fluorescent. Scale bar = 100 um. (b) Apoptosis rate was calculated by IPP software from five visual fields in each group. Apoptosis rate declined significantly in DSS group. (c) Western blot results of caspase-3 protein expression. (d) Statistic data of caspase-3 protein expression. Values were expressed as mean ± SEM. ^*∗*^*P* < 0.05, ^*∗∗*^*P* < 0.01, compared to control group. ^#^*P* < 0.05, ^##^*P* < 0.01, compared to model group.

**Figure 4:** (a) Mitochondrial membrane potential (MMP) was detected by JC-1 dye. MMP declined significantly in model group and remained normal level in DSS group. (b) Mitochondrion permeability transition pore (MPTP) was detected by MPTP kit. RFU decline means MPTP opening degree upregulated. Thus, MPTP opening significantly upregulated in model group but not in DSS group. Values were expressed as mean ± SEM. ^*∗*^*P* < 0.05, compared to control group. ^#^*P* < 0.05, compared to model group.

**Figure 5:** *ATP 5G1 expression*. (a) ATP 5G1 mRNA expression was detected by QPCR. (b) Western blot results of ATP 5G1 protein expression. (c) Statistic data of ATP 5G1 protein expression. Values were expressed as mean ± SEM. ^*∗∗*^*P* < 0.01, compared to control group. ^##^*P* < 0.01, compared to model group.

**Figure 6:** *Cell experiments*. (a-b) Transfection effect evaluation: (a) ATP 5G1 mRNA expression detected by QPCR after transfection experiment. (b) ATP 5G1 protein expression detected by western blotting after transfection experiment. (c) Statistic data of ATP 5G1 protein expression after transfection experiment. (d) Cell viability detected by CCK-8. (e) ATP 5G1 mRNA expression in each group. (f) MPTP opening detected by MPTP kit. Values were expressed as mean ± SEM. ^*∗*^*P* < 0.05, ^*∗∗*^*P* < 0.01, compared to control group. ^#^*P* < 0.05, compared to model group.

The article "Cardioprotective Effect of Danshensu against Ischemic/Reperfusion Injury via c-Subunit of ATP Synthase Inhibition" was published in 2017. Journal: Evid Based Complement Alternat Med.

**Figure 7:** *Cell apoptosis rate detected by TUNEL and DAPI*. Nuclear was stained by DAPI and presents blue fluorescent. Apoptosis was detected by DNA strand breaks stained by TUNEL kit and presents green fluorescent. Scale bar = 50 um. Values were expressed as mean ± SEM. ^*∗∗*^*P* < 0.05, compared to control group. ^##^*P* < 0.01, compared to model group.
